The article "Locomotion Mode Recognition with Inertial Signals for Hip Joint Exoskeleton" was published in 2021. Journal: Appl Bionics Biomech.

# Locomotion Mode Recognition with Inertial Signals for Hip Joint Exoskeleton

**DOI:** 10.1155/2021/6673018

**Published:** 2021-05-24

**Authors:** Gang Du, Jinchen Zeng, Cheng Gong, Enhao Zheng

**Affiliations:** ^1^School of Information Engineering, China University of Geosciences, Beijing 100083, China; ^2^Faculty of Electrical Engineering, Mathematics and Computer Science, Technische Universiteit Delft, Delft 2600AA, Netherlands; ^3^College of Engineering, Peking University, Beijing 100871, China; ^4^The State Key Laboratory of Management and Control for Complex Systems, Institute of Automation, Chinese Academy of Sciences, Beijing 100190, China

## Abstract

Recognizing locomotion modes is a crucial step in controlling lower-limb exoskeletons/orthoses. Our study proposed a fuzzy-logic-based locomotion mode/transition recognition approach that uses the onrobot inertial sensors for a hip joint exoskeleton (active pelvic orthosis). The method outputs the recognition decisions at each extreme point of the hip joint angles purely relying on the integrated inertial sensors. Compared with the related studies, our approach enables calibrations and recognition without additional sensors on the feet. We validated the method by measuring four locomotion modes and eight locomotion transitions on three able-bodied subjects wearing an active pelvic orthosis (APO). The average recognition accuracy was 92.46% for intrasubject crossvalidation and 93.16% for intersubject crossvalidation. The average time delay during the transitions was 1897.9 ms (28.95% one gait cycle). The results were at the same level as the related studies. On the other side, the study is limited in the small sample size of the subjects, and the results are preliminary. Future efforts will be paid on more extensive evaluations in practical applications.

## 1. Introduction

Lower-limb exoskeletons/orthoses serve as important roles in rehabilitation, industrial manufacture, and other human-centered areas [1]. The specifically designed mechanical structures and the control strategies can alleviate the loads on the human body and thus increase the wearer's absolute strength in heavy load bearing or endurance in long-term tasks. There are various types of exoskeletons according to the active joints, such as whole-body exoskeletons (e.g., BLEEX [2] and HAL [3]) and single-joint ones [4] (e.g., hip joint and ankle joint). The hip joint connects the lower extremity and the trunk. The hip joint's primary function is to support the weight of the body in both static (e.g., standing) and dynamic (e.g., walking) postures [5]. The development of the hip joint exoskeleton is a hot research topic in this area. There are many groups developing hip joint exoskeletons (or active pelvic orthoses) all over the world [6–13]. The assistance on the hip joint helps to stabilize the locomotion [6–9], optimize the metabolic cost [10, 11], adjust the abnormal gait patterns [12], and reduce the extra loads on the spine [13], according to the design of the exoskeleton.

The article "Locomotion Mode Recognition with Inertial Signals for Hip Joint Exoskeleton" was published in 2021. Journal: Appl Bionics Biomech.

One primary step in exoskeleton control is to recognize lower-limb motion intents accurately. It bridges the gap between the human sensorimotor system and the external robotic controllers, the performance of which determines the safety and working efficiency of the whole system [4]. The recognition tasks include gait phase estimation/detection, locomotion mode recognition, and other joint motion parameter estimations. Locomotion mode recognition involves the ambulation modes on different terrains (e.g., level ground and stairs) and the nongait patterns (e.g., standing). The recognition system should recognize the current modes and mode transitions accurately on multiple subjects. The recognition approach comprises the sensing system and the processing algorithms. The processing algorithms are usually designed based on the signal features of the sensing system. Previous studies on this area suggest that the neural-mechanical signal fusion method can produce satisfactory recognition results (e.g., accuracies and time latency). The neural signals are usually measured from the muscle signals (e.g., electric activities represented as surface EMG or shape changes represented by the noncontact capacitive sensors). The mechanical signals are measured from the inertial measurement units (IMUs) and loadcell sensors. The sensor nodes can be integrated into the mechanical structure of the exoskeletons. The muscle signals respond faster than the mechanical signals. However, they convey more noises, and the mechanical signals can produce signals with high repeatability due to the advancement of sensing technology. The combination of the signals can compensate each other to get better performance.

The target for locomotion mode recognition is to produce an accuracy as high as possible with the least intervention on the human body. The muscle signals require additional electrodes or front-ends on the human body, which decreases the convenience and the potential willingness of uses. Another limitation is that the recognition parameters should be calibrated for each individual, increasing the time needed before use. For hip joint exoskeleton control, many researchers purely used mechanical signals for human locomotion mode recognition. For instance, the study [14] combined the IMU sensors on an active pelvic orthosis and the foot pressure sensors for gait mode recognition. The designed algorithm was an event-based fuzzy-logic structure triggered by the foot pressure sensors. The study [15] identified different gait modes with the hip joint angles measured from the encoder of the hip joint exoskeleton. The designed algorithm was a multilayer perceptron neural network. The study [14] conducted a real-time locomotion mode recognition with IMU signals when wearing the active pelvic orthosis (APO [8]). The machine learning-based algorithms were trained and tested onboard. The studies mentioned above produced accurate recognition results on various locomotion mode tasks. However, for hip joint exoskeleton control, burdensome calibration for different individuals and additional sensor nodes on the human body still limited practical applications. For instance, the study overcame the subject-dependent problems with sEMG signals, but the system still required pressure insoles on feet to provide gait event information. The study of our group validated the recognition method with the APO. However, subject-dependent training and calibration were needed before testing procedures.

The article "Locomotion Mode Recognition with Inertial Signals for Hip Joint Exoskeleton" was published in 2021. Journal: Appl Bionics Biomech.

In this study, we proposed a locomotion mode recognition method based on inertial measurement unit sensors on the hip joint exoskeleton. The designed fuzzy-logic-based algorithm can overcome the subject-dependent parameters in data training, which does not require training for each subject before uses. Besides, no additional sensors are required on the human body, increasing the convenience in practical applications. We preliminarily evaluated the proposed method with an APO on the locomotion mode and locomotion transition recognition on multiple subjects.

## 2. Experimental Setups

### 2.1. Hip Joint Exoskeleton

In this study, we used an active pelvic orthosis (APO) developed by the research group of Scuola Superiore Sant'Anna (SSSA) [8]. The lightweight exoskeleton can provide assistive torque in the sagittal plane to the hip joints (see Figure 1). The APO was designed with a serial elastic structure based on torsional springs, and the torque was transmitted to the joints with two lightweight carbon fiber-made links (driving part in Figure 1). A C-shaped (in the coronal plane) structure combined with the bandages fixed the exoskeleton to the waist and pelvis of the user, keeping it stable on the human body. Two orthotic shells were connected to the carbon fiber-made links and fixed on the thighs with bandages. The torque was applied to the human body through the shells. There were 3 degree-of-freedoms (DoFs) for each leg, two passive (hip adduction/abduction and pelvic tilting), and one active (flexion/extension) [8]. The passive DoFs ensured the stability of the whole system during ambulation. The core of the actuation system of APO was the DC motors with gearboxes (80 : 1 reduction ratio). The torsional spring was placed on the axis of the flexion/extension of the exoskeleton, between the DC motor (gearbox) and the carbon fiber-made link. The basic calculation of the interaction torque was achieved by the torsional spring constant and the relative position of the encoders [8]. The interaction torques between the human body and the exoskeleton lead to the deformation of the spring. With the integrated encoders and the stiffness of the torsional spring, the control system of the APO can calculate the interaction torques between the human body and the DC motor.

The article "Locomotion Mode Recognition with Inertial Signals for Hip Joint Exoskeleton" was published in 2021. Journal: Appl Bionics Biomech.

The control strategy of APO was hierarchical control. The low-level controller was the torque control. The interaction torques calculated from the encoders served as the feedback of the control loop. The control output determined the applied torque on the human body. There were zero-torque mode and assistive-torque mode. For the zero-torque mode, the desired interaction torques between the legs and the exoskeleton were zero. In the assistive-torque mode, the controller's commanded torque was a predefined curve (in one stride). The high-level controller was an adaptive oscillator- (AOs-) based controller, which used a set of adaptive oscillators to track the phase of one gait cycle continuously. The input of the AO-based controller was the encoder signals representing the hip joint angle information, and the output of the controller was the gait phase at time *t* and the corresponding anticipated torque. One merit of the AO-based controller was the continuous estimation of gait phases with robustness to different walking speeds [16].

### 2.2. Sensing System

We implemented an IMU board on each leg (see Figure 1). The raw signals of the IMU board included 3-axis accelerations and 3-axis gyroscopes. There was a microcontrol unit (MCU) on the board, i.e., ATMEGA328. The MCU calculated the pitch angle and the roll angle (global frame of the Cartesian system) with the acceleration and gyroscope signals. The board was fixed on the cuff of the exoskeleton through a connector (3D printed). The pitch angle of the IMU corresponded to the flexion/extension of the hip joint. The update rate of the tilt angles was 100 Hz.

The data of the IMU boards were transmitted to a control circuit on the back of APO. The control circuit synchronized the data of APO and the IMU boards via Universal Synchronous Asynchronous Receiver Transmitter (USART). The control circuit integrated a WIFI module. The data of the IMU sensors and the states of APO were transmitted to a host computer wirelessly in each 10 ms. A graphic user interface on the computer was designed with MATLAB R2016b to control the data sequence and store the data.

The article "Locomotion Mode Recognition with Inertial Signals for Hip Joint Exoskeleton" was published in 2021. Journal: Appl Bionics Biomech.

### 2.3. Experimental Protocol

In this study, we recruited three healthy subjects. They had an average age of 27.3 years, an average height of 173.7 cm, and an average weight of 67.3 kg. Each subject wore the APO, as shown in Figure 1 in the experiment. In this experiment, we recorded 5 locomotion modes and 8 locomotion transitions. The locomotion modes included standing (St), level walking (LW), stairs ascending (SA), and stairs descending (SD). The locomotion transitions included St⟵⟶LW, LW⟵⟶SA, and LW⟵⟶SD. Each subject performed 4 tasks of ambulation to cover all the locomotion modes and transitions (see Figure 2). For task 1, there were 2 stride cycles of LW and 7 stride cycles of SA (St⟶LW⟶SA⟶St). For task 2, there were 7 stride cycles of SD and 2 stride cycles of LW (St⟶SD⟶LW⟶St). For task 3, there were 3 stride cycles of LW and 5 stride cycles of SD (St⟶LW⟶SD⟶St). For task 4, there were 5 stride cycles of SA and 3 stride cycles of LW (St⟶SA⟶LW⟶St). The tasks in the experiments were shown in Figure 2. The number of stride cycles was shown in Table 1. In our study, to mimic the locomotion in daily activities, we allowed the subjects to perform the locomotion modes at their favorite paces. Therefore, the number of gait cycles of the subjects was different. Three subjects performed different task repetitions. Subject 1 performed 9 repetitions for each task, including LW with 90 gait cycles, SA with 108 gait cycles, SD with 108 gait cycles, and 9 repetitions for each locomotion transition (LW⟶SA, SA⟶LW, gait initiation/termination). Subject 2 performed 5 repetitions for each task, including LW with 50 gait cycles, SA with 60 gait cycles, SD with 60 gait cycles, and 5 repetitions for each locomotion transition. Subject 3 performed 6 repetitions for each task, including LW with 60 gait cycles, SA with 72 gait cycles, SD with 72 gait cycles, and 6 repetitions for each locomotion transition.

## 3. Recognition Method

### 3.1. Cascaded Recognition Method

The locomotion recognition method was designed based on the signal features acquired in the IMUs of both legs. The recognition method is cascaded, which firstly (first layer) classifies the static mode (St) and dynamic modes (LW, SA, SD) and secondly (second layer) identifies the corresponding dynamic locomotion modes (see Figure 3). In the second layer, we designed a fuzzy-logic-based algorithm. There were two membership function sets in the fuzzy-logic-based algorithms, one for each leg. The input of the membership functions was the data pair of peak-valley values detected from the thigh angles. Therefore, in the second layer, we firstly identified the peaks and valleys and secondly calculated the fuzzy-logic membership functions. During the locomotion transitions, there are different leading legs. The procedures of two legs worked independently in the recognition process.

The article "Locomotion Mode Recognition with Inertial Signals for Hip Joint Exoskeleton" was published in 2021. Journal: Appl Bionics Biomech.

In the cascaded recognition method, the first step is to distinguish between the static locomotion mode and the dynamic modes. As there were no gait patterns during standing, the signal profiles were much different from that of ambulation modes. We extracted time-domain features to represent the signal profiles of standing and other locomotion modes. We firstly segmented the data (pitch angles and accelerations) with a 100 ms (10 samplings) sliding window. We calculated the standard deviation on the windows of the left leg's pitch angles std(*θ*_*L*_) and the sum of absolute values of 3-axis accelerations sum(acc). Additionally, we compared the angular difference of the two legs in the sagittal plane, expressed as *θ*_relative_ = |*θ*_*L*_ − *θ*_*R*_|. *θ*_*R*_ is the right thigh's pitch angle, and *θ*_*L*_ is the left thigh's pitch angle. *θ*_relative_ is the relative pitch angle between the left thigh and right thigh. The first layer recognition was achieved by comparing the threshold-based conditions. The logic was expressed as

(1) $$\begin{array}{c} \text{std}\left(\theta_{L}\right)>{Th}_{\text{std}}\text{or}\left|\theta_{L}-\theta_{\text{init}}\right|>{Th}_{\theta }\text{or}\left|\theta_{R}-\theta_{\text{init}}\right|>{Th}_{\theta }\text{ or }sum\left(acc\right)>{Th}_{\text{Acc}}\text{ and }\theta_{\text{relative}}>\theta_{\text{static}.} \end{array}$$

If the logic condition was satisfied, the mode would be recognized as dynamic modes. Otherwise, it was classified as the static mode (St). *θ*_init_ is the initial pitch angle for both thighs which is close to 0.

In the above logic condition, Th_std_ was the standard deviation threshold for the sliding window which was selected as 0.5°. Th_*θ*_  was the pitch angle threshold for both legs which was selected as 8°. *θ*_static_ was the threshold for the static mode which was selected as 10°. Th_Acc_ was the threshold for acceleration which was chosen as 500.

### 3.2. Detecting the Extreme Values

The second layer was to further separate the data into corresponding dynamic locomotion modes (i.e., LW, SA, and SD). We designed a fuzzy-logic-based algorithm to classify the locomotion modes. Each input was a 2 × 1 vector including the peak and valley of the pitch angles. We designed an algorithm find_peak() to detect the peaks and valleys of the IMU signals. The most recent true peak and valley values found by find_peak() would be put in a 2 × 1 buffer as the input of the subsequent fuzzy-logic-based algorithms. Taking finding the left leg's peak values for example (diagram see Figure 4), we firstly predefined thresholds for peak value Th__peak_ and time interval Th__interval_. *θ*_*L*_(*t*) was the pitch angle of the left leg at time *t*. We used *P*(*i*) to represent the *i*_th_ peak value found in (pseudo) real-time. Secondly, the past 21 samples before time *t* were compared (i.e.,  *θ*_*L*_(*t*), *θ*_*L*_(*t* − 1), ⋯, *θ*_*L*_(*t* − 20)). If *θ*_*L*_(*t* − 10) is larger than all the 10 numbers backward ( *θ*_*L*_(*t* − 20), *θ*_*L*_(*t* − 19), ⋯*θ*_*L*_(*t* − 11) and all the 10 numbers forward ( *θ*_*L*_(*t*), *θ*_*L*_(*t* − 1) ⋯ *θ*_*L*_(*t* − 9)), we set *P*(*i*) = *θ*_*L*_(*t* − 10). If the absolute value of peak value *P*(*i*) minus the initial value of pitch angle *θ*_*L*_(0) was larger than Th__peak_, we would consider the peak value *P*(*i*) as an outlier which would be discarded. Otherwise, the *P*(*i*) would be treated as a peak candidate. Because of the existence of false peak values created by the noise, we compared peak candidate's location location*_P*(*i*) with that of the latest candidate location*_P*(*i-*1). We set the time interval threshold Th__interval_ for two adjacent peak values. If the time interval between these two peak values was smaller than Th__interval_, we would assume that one of the two candidate peak values was false. The candidate with the smaller value was aborted. We set a decision flag for the algorithm. The decision flag would be activated if a true peak and a true valley were detected. The peak-valley pair was then inputted to the subsequent fuzzy-logic-based algorithm, and then the flag would be deactivated. The procedure of detecting valleys and the values of the other leg was the same.

The article "Locomotion Mode Recognition with Inertial Signals for Hip Joint Exoskeleton" was published in 2021. Journal: Appl Bionics Biomech.

### 3.3. Fuzzy-Logic-Based Recognition Method

We designed a fuzzy-logic-based method to separate between the locomotion modes of LW, SA, and SD. As mentioned above, the input of the fuzzy-logic algorithm was a 2-dimensional (2D) vector containing the latest detected peak and valley (one leg), represented as *θp* and *θv*, respectively. The maximum/minimum values revealed the characteristics of different locomotion modes. For instance, the *θp* values of SA were larger than that of LW and SD, as the hip joint angles were larger in flexion when ambulating upward. The valleys of the thigh pitch angles also demonstrated similar features. During the LW and SD mode, *θv* values were at the same level, while they would decrease during the SA mode because the stair-ascending locomotion contains a kicking-back movement in which the hanging leg could reach the lowest pitch angle without the constraint of the stairs. During LW and SD, *θv* would be limited by the ground and the stairs. We visualized the characteristics in Figure 5. The distribution of maximum-minimum of different locomotion modes could be separated apart.

We designed multivariate membership functions to classify the three locomotion modes. The membership function calculates the membership value of the event-based feature belonging to the target mode. The output range of membership is (0,1], where 1 is the maximum membership of the model. The membership functions were calculated in parallel with the signals of two legs. For the signals of each leg, we defined three membership functions, one for each locomotion mode. The function was expressed as

(2) $$\begin{array}{c} f_{i}=\frac{k_{i}}{2\pi {\left|\Sigma_{i}\right|}^{1/2}}e^{-\left[\frac{1}{2}{\left(C_{i}-{\bar{X}}_{i}\right)}^{T}\Sigma_{i}^{-1}\left(C_{i}-{\bar{X}}_{i}\right)\right]},i=1,2,3, \end{array}$$

where *i* denoted the mode's number, *k*_*i*_ was the scale factor, *C*_*i*_ = (*θ*_*pi*_, *θ*_*vi*_)^*T*^ was the input vector including the detected peak and valley, and ${\bar{X}}_{i}={\left(\mu_{pi},\mu_{vi}\right)}^{T}$ was the central point of the membership function. In our study, the point was represented as the mean value of the training data sets. *Σ*_*i*_ was the covariance matrix representing the data distribution. After calculating three membership functions of LW, SA, and SD, respectively, the algorithm proceeded to calculate the maximal membership of the target mode:

(3) $$\begin{array}{c} \text{Target mode}=\arg\underset{i}{\max}\left(f_{i}\right). \end{array}$$

Figure 5 shows that 2-dimensional space three membership functions created three oval shape regions, whose center coordinates were the mean value of three membership functions (${\bar{X}}_{i}$). In our study, the parameters ${\bar{X}}_{i}$ and *Σ*_*i*_ were fitted with the training data set (described in detail below).

### 3.4. Synchronization of the Recognition Decisions

There were inertial sensors on both thighs. The fuzzy-logic-based recognition method worked in parallel for the left leg and the right leg. The recognition decisions were then synchronized to minimize the errors in locomotion transitions. In our cascaded recognition method, the first layer was to distinguish between St and dynamic modes. The transitions were gait initiation and gait termination. For gait initiation recognition (St⟶other modes), the first recognized transition was deemed to be the results, which were expressed as

(4) $$\begin{array}{c} t_{i}=\min\left[\left(\text{right }{\text{legs}}^{\prime }\text{s transition time point }t_{R}\right),\left(\text{left le}{\text{g}}^{\prime }\text{s transition time }t_{L}\right)\right], \end{array}$$

where *t*_*i*_ was the timing point of the detected transition. For gait termination recognition, the last recognized transition was deemed to the recognition results. The timing point *t*_*t*_ was expressed as

(5) $$\begin{array}{c} t_{t}=\max\left[\left(\text{right }{\text{leg}}^{\prime }\text{s transition time point }t_{R}\right),\left(\text{left le}{\text{g}}^{\prime }\text{s transition time }t_{L}\right)\right]. \end{array}$$

For the second layer recognition, the transition timing points (*t*_0*d*_) were the first recognized timing points between the left leg's and right leg's results.

The article "Locomotion Mode Recognition with Inertial Signals for Hip Joint Exoskeleton" was published in 2021. Journal: Appl Bionics Biomech.

## 4. Evaluation Method

### 4.1. Crossvalidation

We used the crossvalidation method to evaluate the performances. We evaluated the performance with 1 : 2 intersubject crossvalidation and 1 : 1 intrasubject crossvalidation. In the 1 : 1 intrasubject crossvalidation, each subject's data were divided into two sets with the same sizes. The first data were used for training, and the second set for testing. The procedure was repeated with the second data set for training and the first set for testing. The results of the two tests were averaged as the result of the subject. In the 1 : 2 intersubject crossvalidation, we used the data of one subject for training and the data of the other subjects for testing. In the training procedure, the parameters of the fuzzy-logic-based algorithms were fitted.

### 4.2. Recognition Accuracy

The first metric for evaluating the performance was the recognition accuracy.

In the first layer, the recognition decisions (St and other dynamic modes) were continuously calculated in each sample. The recognition accuracy (*recognition accuracy* 1) was defined as

(6) $$\begin{array}{c} \text{recognition accuracy}1\left(i\right)=\frac{N\text{correct}1\left(i\right)}{N\text{total}1\left(i\right)}, \end{array}$$

where *i* was the subject's number, *N*correct1 was the number of correctly recognized decisions, and *N*total1 was the total number of decisions.

In the second layer, the recognition decisions were calculated in each extreme point being detected (peak and valley). The recognition accuracy of the second layer was defined as

(7) $$\begin{array}{c} \text{recognition accuracy}\left(i\right)=\frac{N\text{correct}\left(i\right)}{N\text{total}\left(i\right)}, \end{array}$$

where *i* was the number of subjects, *N*correct was the number of correctly recognized gait cycles, and *N*total was the total number of gait cycles.

The article "Locomotion Mode Recognition with Inertial Signals for Hip Joint Exoskeleton" was published in 2021. Journal: Appl Bionics Biomech.

### 4.3. Confusion Matrix

We used the confusion matrix to illustrate the recognition performance of each locomotion mode. The details of the definition can be found in [17].

### 4.4. Time Delay of the Locomotion Transitions

Another metric for evaluating the performance was the time delay. There were three critical timing points in each transition period, i.e., the timing point when the data changed from St to dynamic modes (gait initiation, *t*_0*i*_), the timing point when the data changed from dynamic modes to St (gait termination, *t*_0*t*_), and the timing point when the data changed from one dynamic mode to another (*t*_0*d*_).

The reference transition time was determined by labels. In our cascaded recognition method, the first layer was to separate between standing and dynamic modes. We manually labeled the data as standing and dynamic modes by IMU signals. If the pitch angles exceeded a threshold compared with that of standing, the data would be labeled as dynamic modes, and *t*_0*i*_ was defined as the reference of the gait initiation transition time between standing and dynamic modes, while *t*_0*t*_ was defined as the reference of the gait termination transition time between dynamic and standing modes. For the second layer recognition, the reference transition time was labeled based on the gait events detected by the foot pressure insoles. *t*_0*d*_ was defined as the reference of the transition time between two dynamic modes. *t*_0*d*_ would be labeled as the middle point of the swing phase. The labeling method motion transitions were the same as that of existing-related studies [18, 19].

The time delay (Td_init) of gait initiations was defined as the difference between the recognized timing point *t*_*i*_ and the reference transition time of gait initiation  *t*_0*i*_, expressing as

(8) $$\begin{array}{c} \text{Td\_init}=t_{i}-{\text{t}}_{0i}. \end{array}$$

Similarly, the timed delay (Td_terminal) of gait terminations was expressed as

(9) $$\begin{array}{c} \text{Td\_terminal}=t_{t}-t_{0t}, \end{array}$$

where *t*_*t*_ was the recognition transition time of gait termination, and *t*_0*t*_ was the reference transition time of gait termination.

The time delay (Td_dynamic) of the dynamic modes was expressed as

(10) $$\begin{array}{c} \text{Td\_dynamic}=t_{d}-t_{0d}, \end{array}$$

where *t*_*d*_ was the recognition transition time of dynamic modes, and *t*_0*d*_ was the reference transition time of dynamic modes. The positive value presented the delay of recognition, and the negative value represented the advance of recognition, shown in Figure 6.

## 5. Results

### 5.1. Recognition Accuracy

In this section, we showed the recognition accuracy for both the first and second layer classifiers. The first layer recognition was designed to distinguish dynamic modes from standing (St). The second layer recognition was designed to classify three dynamic modes (LW, SA, and SD).

The article "Locomotion Mode Recognition with Inertial Signals for Hip Joint Exoskeleton" was published in 2021. Journal: Appl Bionics Biomech.

As for the first layer (classification between dynamic modes and St), the recognition accuracy for each subject was 92.18%, 93.00%, and 90.45%, respectively. The average recognition accuracy was 91.88%. As for the second layer (classification between LW, SA, and SD), the fuzzy-logic-based method produced accurate recognition decisions in locomotion mode tasks (the case result see Figure 6). The recognition accuracy was higher than 0.89 for most of the evaluations (intersubject shown in Table 2 and intrasubject shown in Table 3). In Tables 2 and 3, each row represented the subject number used for training, and each column represented the testing data (the subject used for testing). The offdiagonal results in Table 2 were the intersubject recognition accuracies, while the diagonal results in Table 3 denoted the accuracies of the intrasubject crossvalidation.

In the 1 : 2 intersubject validation (see in Table 2), the membership functions trained with subject3's dataset had the best performance, with the highest accuracy, 95.51%. The average recognition accuracy for each subject trained with different datasets was 91.54%, 92.80%, and 95.14% for subject 1, subject 2, and subject 3, respectively. The lowest accuracy (89.84%) occurred in subject 1 trained with subject 2's dataset. Subject 3's average recognition accuracy showed the best performance, 95.14%.

In Table 3 (intrasubject crossvalidation), recognition accuracies showed a similar pattern but slightly decreased compared with intersubject validation. The lowest accuracy, 86.80%, occurred in subject 1 trained with subject3's dataset. The average testing set recognition accuracy of three subjects trained with the same training dataset was 92.98%, 93.26%, and 91.16%, respectively, with subject 1, subject 2, and subject3's training dataset. The average testing set recognition accuracy for each subject trained with different training datasets was 87.62%, 94.27%, and 95.51%, respectively.

In Tables 4 and 5, we presented the recognition accuracy for each task. From the experiment results, the lowest recognition accuracy for each subject's results usually occurred in task 2 (St⟶SD⟶LW⟶St), while the recognition algorithm usually performed better in task 1 and task 4.

### 5.2. Time Delay of Locomotion Transitions

We investigated the time delay during locomotion transitions trained/tested with half the data of a subject. We calculated the time difference between the recognized locomotion transitions and the referenced ones. We defined the time latency of gait initiations as Td_init, gait terminations as Td_terminal, and the dynamic transition as Td_dynamic. The unit of the results was ms.

The article "Locomotion Mode Recognition with Inertial Signals for Hip Joint Exoskeleton" was published in 2021. Journal: Appl Bionics Biomech.

From Table 6, we can see that the average time delay of gait initiations for each subject was 1077.3 ms, 812.8 ms, and 268.2 ms and the average time delay of gait terminations was 787.5 ms, 315.5 ms, and 29.2 ms. The average time delay for all the subjects was 554.4 ms. Subject 3 has the lowest time delay for both gait initiations and gait terminations (268.2 ms and 29.2 ms). Also, we can find that large time delays occurred in task 2 and task 3 frequently.

For Table 7, we can see that the average Td_dynamic for each subject was 685.1 ms, 541.8 ms, and 394.0 ms. The lowest average Td_dynamic also occurred in subject 3. Also, we can see that the large Td_dynamic usually occurred in task 3.

The average gait cycle was 1897.9 ms, for which the average time delay of average Td_init, average Td_terminal, and average Td_dynamic was 549.5 ms accounted for 28.95% of a gait cycle.

## 6. Discussion

### 6.1. Recognition Performances

In this study, we designed and evaluated the fuzzy-logic-based method for locomotion mode/transition recognition with a hip joint exoskeleton. The method only relied on the inertial sensors integrated into the exoskeleton, and no additional sensors were required on the human body. Compared with the previous works using the same exoskeleton [14, 20], one improvement of our current study was that we simplified the setups of the sensing approaches in both training and testing procedures. The simplification in sensors can reduce the time needed to calibrate the recognition procedure in practical applications.

There are many studies on IMU-based locomotion mode recognition. The performances are determined by the factors, including the sensor setups (sensors' number, sensing positions), the robotic devices (exoskeletons, prostheses), and the processing algorithms. The evaluation method also influenced the numeric recognition results. For instance, the recent studies on IMU-based locomotion mode recognition achieved >95% average recognition accuracies with intrasubject crossvalidation [21, 22]. The sensor setups are quite different from ours. The study mounted an IMU board on the amputated foot for terrain identification [21], while the study fixed the IMU boards on the shanks, the waist, and wrists [22].

In our study, the IMU boards were fixed on the thighs of the subjects. The target robot platform is the hip exoskeleton. The recognition performances of our study were at the same level as that of the previous studies with similar sensor/robot setups [14, 20]. In the previous work with the active pelvic orthosis [14], the authors used inertial sensors on the thigh and the foot pressure insoles for seven locomotion mode recognitions. The average accuracies on six healthy subjects achieved over 99% with locomotion transition tasks. The average time delay during the locomotion transitions was fixed to one step. On the other hand, the authors also claimed the limitations of using additional foot insoles which was not integrated on the exoskeleton. The accuracies decreased to 65.7%-91.2% in different testing data sets if the centre-of-pressure (CoP) information was removed [14]. In our previous works [20], the authors designed machine-learning-based algorithms for locomotion mode recognition. In the study of [23], the authors designed an artificial neural network- (ANN-) based recognition algorithm with the inertial signals (thigh) and the foot pressure signals. The average recognition accuracies were over 98% with subject-dependent training and testing processes. The calculation time of each recognition decision was less than 1 ms, but the time delay of locomotion transitions was not reported. By comparison, in our study, we produced an average recognition accuracy of 93.16% with 1 vs. 2 intersubject crossvalidations and 92.46% with 1 vs. 1 intrasubject crossvalidation.

The article "Locomotion Mode Recognition with Inertial Signals for Hip Joint Exoskeleton" was published in 2021. Journal: Appl Bionics Biomech.

### 6.2. Confounding Factors

One key factor that influenced the recognition accuracies was the detection of the peaks and valleys from the inertial signals. As shown in Figure 6, the locomotion modes and transitions were successfully recognized; although, there were misdetections in the extreme values. The output value of the membership functions was determined by the detected values of the extreme points. In the calculated recognition results, the fuzzy-logic-based method could successfully tell apart the locomotion modes as long as the distribution of the extreme points was distinguishable (as shown in Figure 5). In our study, although no signals from the feet were measured, the maximum/minimum angles still showed gait information. The maximum value of the thigh tilt angle usually occurred at the swing phase, which was used to distinguish between the LW and SA. While the minimum angle occurred near the foot-off of one gait cycle, the values were informative to distinguish between LW and SD. The maximum hip flexion/extension angles are highly correlated to the locomotion modes. For instance, the maximum flexion angles of SA were significantly larger than that of LW and SD. The subjects can adjust the patterns intuitively to control the exoskeletons in locomotion transition tasks. The physical significance of the features in our fuzzy-logic-based algorithm can accelerate the training/calibration procedure for a novice subject. Another point worth being noted is the intersubject variability in signal profiles and recognition performances. In addition to the difference in motion patterns, the difference in relative positions of the IMU boards on the thigh was another important reason. During the experiments, the IMU boards were fixed on the same positions at the exoskeleton. Due to the different anthropometries of the subjects, the relative positions on the thigh were different. In practical applications, the sensors usually are fixed on the exoskeleton. Adjusting the sensor position to keep the same signal profiles across subjects is also impractical. In future real-time control, we will improve the recognition algorithms with the ability of fast calibration to make the trained model quickly update with the new user.

The article "Locomotion Mode Recognition with Inertial Signals for Hip Joint Exoskeleton" was published in 2021. Journal: Appl Bionics Biomech.

### 6.3. Influence of the Recognition Performances on Robotic Control

In real-time control of the APO, the hierarchical control framework is usually designed. The high-level controller recognizes the locomotion modes and determines the assistive torque curve of the recognized terrain. The middle-level controller uses adaptive oscillators (AOs) to track the desired torque curve. The low-level controller drives the motors to achieve the force feedback loop.

If there are recognition errors, the desired torque curve for the controller will be different from that needed for the current terrain. The user will move with an inappropriate assistive torque curve. The APO applies assistive torque on the hip joint angle in the sagittal plane. Due to the mechanical design of the APO (2 passive DoFs in the coronal plane and passive compliance), it is less likely that the user will fall caused by the wrong recognition of the locomotion modes. However, in the long-time use, the mismatching between the assistive torque curve and the terrains can increase the metabolic cost (decrease the efficacy of the exoskeleton) and the risks of the fall. If the transition time delay exceeds the starting timing point of the applied assistive torque of one stride, there will be a mismatch between the assistance and the actual locomotion mode. Otherwise, the time delay is acceptable. In our study, the average time delay during the transitions ranges from 300 ms to 1000 ms, which can cause a mismatch between the assistive torques and current locomotion modes. The impacts on the user are the same as that of the recognition errors.

To quantitatively evaluate the recognition errors, further extensive experiments combing the real-time recognition and exoskeleton controller are needed. In future studies, we will investigate the effects of the errors and time delay with real-time recognition and control.

The article "Locomotion Mode Recognition with Inertial Signals for Hip Joint Exoskeleton" was published in 2021. Journal: Appl Bionics Biomech.

### 6.4. Limitations and Future Works

Our current study has some limitations, and the following issues will be addressed in future works. Firstly, the sample size of the subjects was small (*N* = 3). The results were calculated with an offline evaluation. The generalization ability of the fuzzy-logic-based algorithm cannot be extensively evaluated with the small sample size. Due to the individual difference in locomotion patterns and sensor placements, the signal profiles can vary across the subjects. The onboard training and real-time exoskeleton control have yet to be studied. In future works, we will carry out an extensive study on real-time control with onboard training. We will investigate the effects of false detections on control performances. We will also carry out experiments on more subjects to evaluate the generalization performances. Postprocessing approaches will also be designed to remove the recognition errors further. Secondly, the recognition tasks in our study only involved structured terrains in the laboratory environment. In future works, more complicated tasks, including various walking speeds, jogging, and other locomotion modes in daily life, will be investigated. Thirdly, the recognition decisions in our study were discrete in one gait cycle. In future works, we will investigate continuous parameter changes in the locomotion tasks, such as different heights of stairs and different upward locomotion modes (ramps and stairs). The processing algorithm will also be studied to cope with more complicated problems.

## 7. Conclusions

In this study, we designed and preliminarily validated the feasibility of a fuzzy-logic-based algorithm for the locomotion mode and locomotion transition recognition with an active pelvic orthosis. The method purely relied on the inertial signals measured from the thigh, and the sensors were fixed on the exoskeleton. With a proper training process, the fuzzy-based algorithm produced comparable recognition accuracies to the existing studies on the same robotic platform. The superiority of the method was that it required no additional sensors on the human body, increasing the convenience in practical applications. The inputs of the fuzzy-logic-based method were the detected peaks and valleys of the pitch angles of the thigh. Combined with the cascaded recognition method, it produced reliable recognition results as long as the detected extreme points were distinguishable between the dynamic locomotion modes. Future works will be focused on onboard training and real-time control of the exoskeleton, investigation of the complicated unstructured terrains, and adaptation to continuous ambulation parameters.

The article "Locomotion Mode Recognition with Inertial Signals for Hip Joint Exoskeleton" was published in 2021. Journal: Appl Bionics Biomech.

## Figures and Tables

**Figure 1:** The hardware of the system, including the active pelvic orthosis (APO) and the IMU for measurement.

**Figure 2:** The tasks in the experiments. St denotes standing, LW is short for level walking, SA is short for stair ascending, and SD is short for stair descending. The arrows indicate ambulation direction. The tasks are denoted with different colors.

**Figure 3:** The diagram of the recognition method. The first layer was to distinguish dynamic modes from standing (St). The second layer was designed to classify the dynamic modes, and there were three dynamic modes (LW, SA, and SD).

**Figure 4:** The flow chart of finding a peak value from the thigh pitch angles.

**Figure 5:** The distribution of the data of LW, SA, and SD (denoted by the dots) and the calculated membership function (represented by the ellipses). The data of LW, SA, and SD were represented as the yellow dots, the red dots, and the blue dots, respectively. The data were collected from subject 1.

**Figure 6:** The pseudo real-time recognition decisions. The upper subplot is the raw pitch angles and the detected extreme points. The bottom subplot shows the recognition decisions and the reference labels.

**Table 1:** The stride cycle number in each task.

	Task 1	Task 2	Task 3	Task 4
LW (stride)	2	2	3	3
SA (stride)	7	0	0	5
SD (stride)	0	7	5	0

**Table 2:** Training/testing with whole data of a subject (1 : 2 intersubject validation).

	Subject 1	Subject 2	Subject 3
Subject 1	—	90.39%	94.76%
Subject 2	89.84%	—	95.51%
Subject 3	93.23%	95.20%	—

**Table 3:** Training/testing with half data of a subject (1 : 1 intrasubject validation).

	Subject 1	Subject 2	Subject 3
Subject 1	88.29%	95.42%	95.22%
Subject 2	87.76%	95.31%	96.70%
Subject 3	86.80%	92.07%	94.60%

**Table 4:** Recognition accuracy of 1 : 2 intersubject validation.

		Subject 1			Subject 2			Subject 3		
		Number of error steps	Number of total steps	Accuracy rate	Number of error steps	Number of total steps	Accuracy rate	Number of error steps	Number of total steps	Accuracy rate
Subject 1	Task 1	—	—	—	2	95	98.48%	1	109	99.08%
	Task 2	—	—	—	20	85	76.47%	12	102	88.24%
	Task 3	—	—	—	10	74	86.49%	7	93	92.47%
	Task 4	—	—	—	0	82	100.00%	1	97	98.97%

Subject 2	Task 1	15	174	91.38%	—	—	—	1	109	99.08%
	Task 2	21	176	88.07%	—	—	—	10	102	90.20%
	Task 3	18	175	89.71%	—	—	—	6	93	93.55%
	Task 4	15	154	90.26%	—	—	—	1	97	98.97%

Subject 3	Task 1	18	174	89.66%	3	132	97.73%	—	—	—
	Task 2	19	176	89.20%	8	85	90.59%	—	—	—
	Task 3	12	175	93.14%	3	74	95.95%	—	—	—
	Task 4	18	154	88.31%	2	82	97.56%	—	—	—

The article "Locomotion Mode Recognition with Inertial Signals for Hip Joint Exoskeleton" was published in 2021. Journal: Appl Bionics Biomech.

**Table 5:** Recognition accuracy of 1 : 1 intrasubject crossvalidation.

		Subject 1			Subject 2			Subject 3		
		Number of error steps	Number of total steps	Accuracy rate	Number of error steps	Number of total steps	Accuracy rate	Number of error steps	Number of total steps	Accuracy rate
Subject 1	Task 1	1	79	98.73%	1	37	97.30%	0	54	100.00%
	Task 2	15	83	81.93%	5	32	84.38%	6	56	89.29%
	Task 3	18	78	76.92%	0	28	100.00%	3	47	93.62%
	Task 4	3	68	95.59%	0	33	100.00%	1	49	97.96%

Subject 2	Task 1	9	79	88.61%	1	37	97.30%	0	54	100.00%
	Task 2	12	83	85.54%	4	32	87.50%	5	56	91.07%
	Task 3	10	78	87.18%	1	28	96.43%	2	47	95.74%
	Task 4	7	68	89.71%	0	33	100.00%	0	49	100.00%

Subject 3	Task 1	10	79	87.34%	1	37	97.30%	0	54	100.00%
	Task 2	10	83	87.95%	7	32	78.13%	4	56	92.86%
	Task 3	7	78	91.03%	2	28	92.86%	2	47	95.74%
	Task 4	13	68	80.88%	0	33	100.00%	5	49	89.80%

**Table 6:** The initial and terminal transition time latency.

		Subject 1		Subject 2		Subject 3	
		Td_init	Td_teminal	Td_init	Td_teminal	Td_init	Td_teminal
Subject 1	Task 1	—	—	836.0	376.0	-300.0	161.7
	Task 2	—	—	1126.0	-354.0	1145.0	-443.3
	Task 3	—	—	390.0	1626.0	-145.0	-556.0
	Task 4	—	—	376.0	-184.0	-156.0	-527.5

Subject 2	Task 1	2270.0	192.2	—	—	-320.0	235.0
	Task 2	1207.8	-1266.7	—	—	1805.0	-436.7
	Task 3	414.4	2652.2	—	—	-185.0	1768.3
	Task 4	1241.1	641.1	—	—	301.7	31.7

Subject 3	Task 1	567.8	305.6	840.0	334.0	—	—
	Task 2	904.4	764.4	1630.0	110.0	—	—
	Task 3	705.6	2198.9	964.0	452.0	—	—
	Task 4	1307.8	812.2	340.0	452.0	—	—

**Table 7:** The dynamic transition time latency.

		Td_dynamic		
		Subject 1	Subject 2	Subject 3
Subject 1	LW⟶SA	—	444.0	230.0
	SD⟶LW	—	136.0	-405.0
	LW⟶SD	—	1696.0	1815.0
	Sa⟶LW	—	-154.0	-1.7

Subject 2	LW⟶SA	235.6	—	230.0
	SD⟶LW	5.6	—	-405.0
	LW⟶SD	235.6	—	1690.0
	Sa⟶LW	687.8	—	-1.7

Subject 3	LW⟶SA	365.6	444.0	—
	SD⟶LW	921.1	136.0	—
	LW⟶SD	2198.9	1526.0	—
	Sa⟶LW	814.4	106.0	—

## Data Availability

The data are made available through the corresponding authors' emails.
